# Efficacy of Neoadjuvant Chemotherapy plus Limb-Sparing Surgery for Osteosarcoma and Its Impact on Long-Term Quality of Life

**DOI:** 10.1155/2022/1693824

**Published:** 2022-08-08

**Authors:** Shixia Jing, Fengling Ding, Yinghong Yuan, Jing An, Qiang He

**Affiliations:** ^1^Central Sterile Supply Department, Nanchong Central Hospital, Nanchong 637000, China; ^2^Department of Orthopedics, Rizhao Central Hospital, Rizhao 276800, China; ^3^Department of Surgery, Nanchong Central Hospital, Nanchong 637000, China; ^4^Department of Infectious Diseases, Rizhao Central Hospital, Rizhao 276800, China; ^5^The Affifiliated Nanhua Hospital, Department of Hand Surgery, Hengyang Medical School, University of South China, Hengyang, Hunan 421001, China

## Abstract

**Purpose:**

To assess the efficacy of neoadjuvant chemotherapy plus limb-sparing surgery for osteosarcoma and its impact on long-term quality of life.

**Methods:**

Between August 2016 and December 2018, 90 patients with osteosarcoma treated in Nanchong Central Hospital were recruited and divided at a ratio of 1 : 1 to receive limb-sparing surgery (control group) or limb-sparing surgery plus neoadjuvant chemotherapy (study group) by random number table methods. The clinical endpoints were clinical efficacy and long-term quality of life.

**Results:**

Limb-sparing surgery plus neoadjuvant chemotherapy was associated with a significantly higher efficacy versus limb-sparing surgery alone. Limb-sparing surgery plus neoadjuvant chemotherapy resulted in a significantly higher Enneking score and a higher good function rating of patients versus limb-sparing surgery. The two groups showed a high but similar 1-year survival rate. Patients given limb-sparing surgery plus neoadjuvant chemotherapy showed significantly higher 2-year and 3-year survival and a longer mean survival versus those receiving limb-sparing surgery alone. Limb-sparing surgery plus neoadjuvant chemotherapy resulted in significantly higher scores of role emotional, mental health, physical function, and social function and a lower bodily pain score than limb-sparing surgery alone. Limb-sparing surgery plus neoadjuvant chemotherapy was associated with significantly lower fatigue, nausea and vomiting, dyspnea, constipation, and diarrhea scores and a significantly higher health status score versus monotherapy of limb-sparing surgery.

**Conclusion:**

Neoadjuvant chemotherapy plus limb-sparing surgery improves the postoperative limb function and long-term quality of life of patients with osteosarcoma, which shows great potential for clinical promotion.

## 1. Introduction

Osteosarcoma is a common malignant bone tumor with an annual incidence of about 4-5 per one million people as reported by epidemiological statistics [1, 2]. The main clinical symptoms are skeletal and joint pain with progressive exacerbation, accompanied by local masses and venous rage. The male-to-female incidence ratio of osteosarcoma is approximately 3 : 2, with approximately 60% of patients with osteosarcoma being under 25 years of age [3, 4]. The most involved body parts are the distal femur, proximal tibia, and the medullary end of the proximal humerus. Clinical reports indicate that osteosarcoma is associated with complications such as pain, tissue remission, limited joint motion, and muscle atrophy, which may severely compromise prognosis and threaten patients' lives. The mortality of the disease remains at a high level despite early and timely treatment [5]. Pathological findings show that osteosarcoma is highly malignant, and the closer the tumor site is to the trunk, the poorer the long-term survival of patients [6].

Radical surgery is indicated for the treatment of osteosarcoma, and limb-sparing surgery is currently considered a promising treatment method. Limb-preserving surgery [7] is a highly specialized procedure that requires extensive tumor resection as per the principles of the surgical management of bone tumors, and postoperative consolidation chemotherapy or radiotherapy is mostly adopted to control tumor metastasis and improve patient survival [8, 9]. Most osteosarcomas of the extremities can be surgically saved. Generally, after neoadjuvant chemotherapy, surgery is performed to save limbs. The 5-year survival rate of common osteosarcoma can reach about 65%. The key technique of limb salvage for osteosarcoma is to ensure clean surgical resection and limb preservation. General surgical methods include prosthesis replacement, allogeneic bone replacement, and reconstruction. Neoadjuvant chemotherapy [10] is a systemic chemotherapeutic approach to minimize tumor size and eliminate invisible metastatic cells to facilitate subsequent treatment [11]. It has been suggested that neoadjuvant chemotherapy combined with limb-sparing surgery is the ideal approach for osteosarcoma [12]. Limb-sparing surgery is a procedure for complete tumor removal without amputation, which is mostly followed by continuous chemotherapy to achieve a satisfactory outcome [13]. Neoadjuvant chemotherapy is systemic chemotherapy administered prior to surgery and provides a favorable foundation for surgery [14]. Neoadjuvant chemotherapy plus surgery is an emerging and effective strategy for the treatment of various cancers, which effectively improves patient prognosis and survival rates [15]. However, there is insufficient clinical evidence for the enrichments in the prognosis and 5-year survival by the combination of neoadjuvant chemotherapy plus limb-sparing surgery. Accordingly, this study was conducted to assess the efficacy of neoadjuvant chemotherapy plus limb-sparing surgery for osteosarcoma and its impact on long-term quality of life, so as to provide relevant references for clinical research.

## 2. Materials and Methods

### 2.1. Research Subjects

In this prospective, randomized, controlled, single-blinded trial, 90 patients with osteosarcoma treated in Nanchong Central Hospital between August 2016 and December 2018 were recruited and divided at a ratio of 1 : 1 to receive limb-sparing surgery (control group) or limb-sparing surgery plus neoadjuvant chemotherapy (study group) by random number table methods. Both patients and family members voluntarily signed the consent form. This study was ethically approved by the Ethical Committee of Nanchong Central Hospital (No. 2016/12-335).

### 2.2. Inclusion and Exclusion Criteria

Inclusion criteria: patients aged 18–70 years, with a diagnosis of osteosarcoma of limbs confirmed by imaging and pathological examination, with stage IIA-IIB (Enneking stage), and with an expected survival of more than one year were included.

Exclusion criteria: patients with heart, liver, kidney, and other vital organ insufficiencies, with relevant contraindications to treatment, and with metastases by the time of diagnosis were excluded.

### 2.3. Treatment Methods

Patients in the control group were treated with limb-sparing surgery and given conventional adjuvant chemotherapy postoperatively.

Limb-sparing surgery: complete extraperitoneal resection (incision margin at least 5 cm from the tumor) [9] was performed, and the necrosis rate of the resected tumor was assessed postoperatively. Patients with a necrosis rate ≥90% were treated with the same chemotherapy regimen and dose of postoperative adjuvant chemotherapy, and patients with a necrosis rate <90% were treated with salvage chemotherapy at an appropriate dose. The duration of postoperative conventional adjuvant chemotherapy was 4 cycles.

Patients in the study group were treated with neoadjuvant chemotherapy plus limb-sparing surgery as follows: after diagnosis, adequate hydration and diuresis were performed 1 day before chemotherapy. The patients received neoadjuvant chemotherapy using the epirubicin (EPI) + cisplatin (DDP) + methotrexate (MTX) + ifosfamide (IFO) regimen. They received 90 mg/m^2^ of EPI on days 1–3, 100 mg/m^2^ of DDP on day 1, and 10 mg/m^2^ of MTX on days 4–10. Each drip was completed within 6 h, followed by 1 dose (15000 mg/m^2^) of calcium folinic acid through intravenous injection every 6 h for a total of 12 doses. On days 15–19, IFO 2000 mg/m^2^ was administered intravenously, and the drip was completed within 6 h, followed by an additional intravenous dose of a-mercapto ethane sulfonic acid sodium salt 400 mg every 6 h for 3 times, as shown in Figure 1. A total of 2 cycles of chemotherapy were administered with 21 days as 1 cycle. After the completion of chemotherapy, limb-sparing surgery was performed, and the surgical procedures were the same as those in the control group. Postoperative chemotherapy was administered in 4 cycles, similar to preoperative chemotherapy.

### 2.4. Outcome Measures

1. Clinical efficacy: the clinical efficacy was evaluated according to the neoadjuvant chemotherapy efficacy assessment criteria, which were classified as complete response (CR), partial response (PR), and progressive disease (PD). CR: patients' symptoms were significantly reduced or disappeared. PR: patients' symptoms were reduced. PD: patients' clinical symptoms were unrelieved.
2. Limb function: six months after treatment, the postoperative functional assessment criteria of Enneking limb musculoskeletal system tumor surgical reconstruction were used to evaluate the limb activity function of the two groups, respectively. The evaluation was performed with regard to six aspects, namely, muscle strength, psychological tolerance, joint mobility, pain, limb stability, and living ability, with 5 points for each item. The postoperative functional assessment grading standard was divided into four levels: excellent, good, moderate, and poor, with ≥24 points as excellent, 18–23 points as good, 12–17 points as moderate, and ≤12 points as poor.
3. Survival: patients were followed up at home or by telephone for 3 years, and the survival of the two groups was recorded and compared separately.
4. Quality of life: six months after treatment, the MOS 36-item short-form health survey (SF-36) health measurement scale was used to assess the patients' quality of life, and the modified quality of life measurement scale for cancer patients (EortcQLQC.30) was used to assess the symptoms and health status of the two groups.

### 2.5. Statistical Analysis

SPSS 22.0 was used for data analyses, and GraphPad Prism 8 was used for image rendering. The measurement data were expressed as ( *x̅* ± *s*) and processed using the *t*-test. The count data were expressed as the number of cases (rate) and analyzed using the chi-square test. Differences were considered statistically significant at *P* < 0.05.

## 3. Results

### 3.1. Baseline Data

In the control group, there were 27 males and 18 females, aged between 19 and 45 (29.88 ± 5.23) years old, with a Karnofsky Performance Scale (KPS) score of 71.62 ± 5.33 points and a maximum tumor diameter of 6.02 ± 1.74 cm. There were 19 cases of the femur, 16 cases of the tibia, and 10 cases of the humerus in terms of tumor sites. In the study group, there were 25 males and 20 females, aged between 20 and 43 (29.94 ± 5.82) years old, with a KPS score of 72.01 ± 4.96 points and a maximum tumor diameter of 5.74 ± 1.93 cm. There were 21 cases of the femur, 15 cases of the tibia, and 9 cases of the humerus in terms of tumor sites. The baseline data of the two groups were comparable (all *P* > 0.05) (Table 1).

### 3.2. Clinical Efficacy

In the control group, there were 14 (31.11%) cases of CR, 21 (46.67%) cases of PR, and 10 (22.22%) cases of PD, with the efficacy of 77.78%. In the study group, there were 21 (46.67%) cases of CR, 22 (48.89%) cases of PR, and 2 (4.44%) cases of PD. Limb-sparing surgery plus neoadjuvant chemotherapy was associated with a significantly higher efficacy versus limb-sparing surgery alone (*P* < 0.05) (Table 2).

### 3.3. Limb Function

Limb-sparing surgery plus neoadjuvant chemotherapy resulted in a significantly higher Enneking score (25.98 ± 3.17 vs. 24.23 ± 2.81) and a higher good function rating result (82.22%, including 21 cases of excellent, 16 cases of good, 5 cases of moderate, and 3 cases of poor) versus limb-sparing surgery (57.78%, including 15 cases of excellent, 11 cases of good, 9 cases of moderate, and 10 cases of poor) (*P* < 0.05) (Table 3).

### 3.4. Survival

The two groups showed a high but similar 1-year survival rate (*P* > 0.05). Patients given limb-sparing surgery plus neoadjuvant chemotherapy showed significantly higher 2-year and 3-year survival and a longer mean survival (91.11%, 84.44%, 33.72 ± 1.08) versus those receiving limb-sparing surgery alone (80.00%, 60.00%, 29.56 ± 0.88) (*P* < 0.05) (Table 4).

### 3.5. Quality of Life

Limb-sparing surgery plus neoadjuvant chemotherapy resulted in significantly higher scores of role emotional, mental health, physical function, and social function and a lower bodily pain score (86.88 ± 7.23, 81.08 ± 5.49, 75.31 ± 6.17, 86.94 ± 3.23, and 62.18 ± 6.77) versus limb-sparing surgery (80.17 ± 6.06, 77.23 ± 5.17, 51.57 ± 6.13, 49.29 ± 8.19, and 70.11 ± 5.84) (*P* < 0.05) (Figure 2). Limb-sparing surgery plus neoadjuvant chemotherapy was associated with significantly lower fatigue, nausea and vomiting, dyspnea, constipation, and diarrhea scores (42.27 ± 4.17, 25.26 ± 3.68, 27.54 ± 3.92, 35.57 ± 2.88, and 25.18 ± 5.07) versus limb-sparing surgery (54.84 ± 4.68, 39.85 ± 4.54, 39.01 ± 4.08, 57.68 ± 5.14, and 39.28 ± 4.17) (*P* < 0.05), and combined therapy also resulted in a significantly higher health status score (67.21 ± 2.34) versus monotherapy (56.88 ± 2.73) (*P* < 0.05) (Table 5).

## 4. Discussion

The results of the present study showed a significantly higher clinical efficacy achieved by limb-sparing surgery plus neoadjuvant chemotherapy (95.56%) versus limb-sparing surgery alone (77.78%). Small metastatic lesions can be mostly unobservable to naked eyes or even imaging, so radical surgery may fail to achieve a satisfactory therapeutic effect. The application of neoadjuvant chemotherapy plays an important role in improving the therapeutic effect and prolonging the survival of patients [16]. The reason for a higher efficacy after combined therapy herein may be that cisplatin is a broad-spectrum anticancer chemotherapeutic agent, which, similar to ifosfamide, acts nonspecifically on the cell division cycle and effectively impedes DNA replication and the expansion and cross-linking of tumor cells to kill cancer cells. Methotrexate is an antifolate antitumor drug that prevents tumor cell synthesis mainly by blocking dihydrofolate reductase inhibition, thereby inhibiting tumor cell growth and regeneration [17].

Osteosarcoma is a relatively drug-resistant tumor, and the effect of single-drug therapy is modest. The combination of antitumor drugs is to kill tumor cells in each cycle, improve the therapeutic effect of patients, and reduce the occurrence of drug resistance [18]. Patients in the present study were required to continue treatment with a chemotherapy regimen after surgical treatment, and the chemotherapy regimen was adjusted according to patients' clinical symptoms to reduce the risk of recurrence and metastasis, which was in line with the findings of Luo et al.[19]. Moreover, in the present study, limb-sparing surgery plus neoadjuvant chemotherapy resulted in significantly higher Enneking scores, good function rating results, 2-year and 3-year survival, mean survival, and quality of life versus limb-sparing surgery alone, suggesting that the use of neoadjuvant chemotherapy combined with limb-sparing surgery was effective in improving patients' limb movement function, survival outcomes, and long-term quality of life. The reason may be that epirubicin directly infiltrates into DNA bases, causing DNA strands to protrude into tumor cells, disrupting the synthesis of DNA and RNA in tumor cells and the structure and function of tumor cell membranes; neoadjuvant chemotherapy reduces the difficulty of surgery and facilitates the successful preservation of limbs [20], thereby enhancing the long-term survival rate and quality of life of patients. However, there are still some shortcomings and deficiencies in this study. The small sample size may compromise the objectivity of the results and conclusions, and only one chemotherapy regimen was proposed in this study, which requires further investigation by future studies.

## 5. Conclusion

Neoadjuvant chemotherapy plus limb-sparing surgery improves the postoperative limb function and long-term quality of life of patients with osteosarcoma, which shows great potential for clinical promotion.

## Figures and Tables

**Figure 1:** Flowchart of neoadjuvant chemotherapy.

**Figure 2:** Comparison of SF-36 scores. ^*∗∗∗*^Difference between the two groups is statistically significant (*P* < 0.001).

**Table 1:** Comparison of baseline data ($\bar{x}$ ± *s*).

	Control group	Study group	*t/χ * ^*2*^	*P*
Gender (male/female)	27/18	25/20	0.182	0.670
Age (years)	29.88 ± 5.23	29.94 ± 5.82	0.51	0.959
KPS scores	71.62 ± 5.33	72.01 ± 4.96	0.359	0.720
Maximum tumor diameter (cm)	6.02 ± 1.74	5.74 ± 1.93	0.723	0.472
Tumor site			0.185	0.912
Femur	19	21		
Tibia	16	15		
Humerus	10	9		

**Table 2:** Comparison of clinical efficacy (%).

Groups	*n*	CR	PR	PD	Efficacy
Control group	45	14 (31.11)	21 (46.67)	10 (22.22)	35 (77.78)
Study group	45	21 (46.67)	22 (48.89)	2 (4.44)	43 (95.56)
*χ * ^2^	—		6.154		
*P*	—		0.013		

**Table 3:** Comparison of limb function.

Groups	*n*	Enneking scores ($\bar{x}$ ± *s*)	Good function rating (*n*, %)
Control group	45	24.23 ± 2.81	26 (57.78)
Study group	45	25.98 ± 3.17	37 (82.22)
*t*/*χ*^2^	—	2.771	6.402
*P*	—	0.007	0.011

**Table 4:** Comparison of survival.

Groups	*n*	1-year survival (*n*, %)	2-year survival (*n*, %)	3-year survival (*n*, %)	Mean survival ($\bar{x}$ ± *s*, month)
Control group	45	41 (91.11)	36 (80.00)	27 (60.00)	29.56 ± 0.88
Study group	45	44 (97.78)	41 (91.11)	38 (84.44)	33.72 ± 1.08
*t/χ * ^2^	—	1.906	3.552	6.702	20.031
*P*	—	0.167	0.049	0.010	<0.001

**Table 5:** Comparison of symptoms and health status ($\bar{x}$ ± *s*).

Groups		Control group (*n* = 45)	Study group (*n* = 45)	*t*	*P*
Symptoms	Fatigue	54.84 ± 4.68	42.27 ± 4.17	13.452	<0.001
	Nausea and vomiting	39.85 ± 4.54	25.26 ± 3.68	16.747	<0.001
	Pain	25.84 ± 3.54	25.68 ± 4.11	0.198	0.843
	Difficulty in breathing	39.01 ± 4.08	27.54 ± 3.92	13.599	<0.001
	Loss of appetite	38.27 ± 3.65	38.44 ± 3.47	0.226	0.822
	Constipation	57.68 ± 5.14	35.57 ± 2.88	25.173	<0.001
	Diarrhea	39.28 ± 4.17	25.18 ± 5.07	14.408	<0.001
Health status	56.88 ± 2.73	67.21 ± 2.34	19.272	<0.001	

## Data Availability

The data generated or analyzed during this study are included within the article.
